RETRACTED

# Stromal interaction molecule 1 regulates growth, cell cycle, and apoptosis of human tongue squamous carcinoma cells

**DOI:** 10.1042/BSR20160519

**Published:** 2017-03-02

**Authors:** Xiaobo Cui, Laixiao Song, Yunfei Bai, Yaping Wang, Boqian Wang, Wei Wang

**Affiliations:** Section of Inner Mongolia Medical University Affiliated Hospital Otorhinolaryngology, Inner Mongolia Medical University Affiliated Hospital, Hohhot, Inner Mongolia 010050, People’s Republic of China

**Keywords:** apoptosis, cell cycle, STIM1, tongue squamous carcinoma, Tca-8113 cells

## Abstract

Oral tongue squamous cell carcinoma (OTSCC) is the most common type of oral carcinomas. However, the molecular mechanism by which OTSCC developed is not fully identified. Stromal interaction molecule 1 (STIM1) is a transmembrane protein, mainly located in the endoplasmic reticulum (ER). STIM1 is involved in several types of cancers. Here, we report that STIM1 contributes to the development of human OTSCC. We knocked down STIM1 in OTSCC cell line Tca-8113 with lentivirus-mediated shRNA and found that STIM1 knockdown repressed the proliferation of Tca-8113 cells. In addition, we also showed that STIM1 deficiency reduced colony number of Tca-8113 cells. Knockdown of STIM1 repressed cells to enter M phase of cell cycle and induced cellular apoptosis. Furthermore, we performed microarray and bioinformatics analysis and found that STIM1 was associated with p53 and MAPK pathways, which may contribute to the effects of STIM1 on cell growth, cell cycle, and apoptosis. Finally, we confirmed that STIM1 controlled the expression of MDM2, cyclin-dependent kinase 4 (CDK4), and growth arrest and DNA damage inducible α (GADD45A) in OTSCC cells. In conclusion, we provide evidence that STIM1 contributes to the development of OTSCC partially through regulating p53 and MAPK pathways to promote cell cycle and survival.

## Introduction

Oral tongue squamous cell carcinoma (OTSCC) is one of the most common cancers diagnosed in the oral cavity comprising 25–40% of oral carcinomas worldwide [1]. This type of cancer is well known for its high rate of lymph nodal metastasis and the number of deaths associated with OTSCC increased during the past 5 years [2]. Despite the identification of some molecular biomarkers for OTSCC, the molecular mechanism underlying OTSCC development remains largely unknown. Identification of novel molecular mechanism will significantly contribute to treatment and prognostic prediction of human OTSCC.

Stromal interaction molecule 1 (STIM1) is a transmembrane protein, mainly located in the endoplasmic reticulum (ER), but also in the plasma membrane, which exhibits an intraluminal region, a single transmembrane segment and a cytoplasmic region [3]. STIM1 is a key component of store-operated calcium entry (SOCE) and plays a dual role as an ER Ca^2+^ receptor and an SOCE exciter. STIM1 senses the ER Ca^2+^ concentration via a luminal, N-terminal located, canonical EF hand. Mutations on the predicted EF hand on residues that are essential for Ca^2+^ binding attenuate the affinity for Ca^2+^ and induce constitutive activation of Ca^2+^ entry even without Ca^2+^ store depletion [4,5].

RETRACTED

STIM1 essentially participates in the development of human cancer by regulating cellular proliferation, cell cycle, apoptosis, and migration [3]. For instance, STIM1 accelerates cell senescence in a remodeled microenvironment but enhances the epithelial-to-mesenchymal transition in prostate cancer [6]. In human hepatocellular carcinoma, STIM1 correlates with elevated hypoxia-inducible factor-1α (HIF-1α) in hypoxic hepatocarcinoma (HCC) cells and is up-regulated in hepatocarcinoma tissues. STIM1-mediated SOCE is required for HIF-1 accumulation in hypoxic HCCs via activation of Ca^2+^/calmodulin-dependent protein kinase II and p300 [6]. In addition, a current report showed that STIM1 promotes tumor metastasis and is associated with poor prognosis in colorectal cancer (CRC) [7]. Our previous work indicated that STIM1 silencing inhibits tumor growth and promotes cell cycle arrest and apoptosis in hypopharyngeal carcinoma [8], indicating that STIM1 may also participate in other types of oral cancers.

In the present study, we report that STIM1 promotes the growth of human OTSCC cells by regulating apoptosis and cell cycle. STIM1 knockdown in OTSCC cells inhibited cellular proliferation and colony formation of cancer cells. We found that STIM1 knockdown repressed cell cycle to enter M phase and induced apoptosis in OSTCC cells. Furthermore, our microarray data showed that STIM1 controlled the p53 and MAPK pathways. Our molecular analysis also confirmed that STIM1 regulated the protein level of MDM2, cyclin-dependent kinase 4 (CDK4), and growth arrest and DNA damage inducible α (GADD45A).

## Materials and methods

### Cell lines and cell culture

The tongue squamous carcinoma cells Tca-8113 were obtained from cell bank of the Chinese Academy of Sciences in Shanghai and cultured in 1640 medium (Sigma–Aldrich, St. Louis, MO, U.S.A.), combined with 10% FBS (Gibco; Thermo Fisher Scientific, Inc., Waltham, MA, U.S.A.) and 1% penicillin/streptomycin (Life Technologies; Thermo Fisher Scientific, Inc.). All the cell cultures were maintained at 37°C in a humid atmosphere containing 5% CO_2_.

### Total mRNA isolation and quantitative real-time PCR

Total RNA was isolated using Trizol reagent (Invitrogen, Carlsbad, CA, U.S.A.) according to the manufacturer’s instructions, and cDNA was synthesized using M-MLV reverse transcriptase (Promega, Shanghai, China). Quantitative real-time PCR (qRT-PCR) was used to analyze STIM1 gene expression using SYBR master mixture (Takara, Tokyo, Japan) on a real-time PCR machine TP800 (Takara, Tokyo, Japan). The relative STIM1 expression was normalized to GAPDH, and data analysis was conducted using the comparative *C*_T_ method. The PCR primers used were as follows: STIM1 forward: 5′-GCCTATATCCAGAACCGTTACTC-3′ and reverse: 5′-TGCTCCAACTCCTCCTCAG-3′, and GAPDH forward: 5′-TGACTTCAACAGCGACACCCA-3′ and reverse: 5′-CACCCTGTTGCTGTAGCCAAA-3′. Cycling conditions for quantitative RT-PCR were as follows: 95°C for 30 s, then 45 cycles of 95°C for 5 s and 60°C for 30 s.

RETRACTED

### Western blot

Total protein was isolated from cultured cells using RIPA lysis buffer (Beyotime, Beijing, China) and then quantitated by the BCA assay kit (Beyotime, Beijing, China). Twenty micrograms of total protein were mixed with 2× loading buffer, separated on SDS/10% PAGE, and then transferred to 0.2 μm PVDF membranes (Millipore, Bedford, MA, U.S.A.). The membranes were blocked in 5% non-fat milk dissolved in TBS and Tween 20 (TBST) buffer for 1 h and incubated with primary antibodies overnight at 4°C. Antibodies against GAPDH (sc-32233, mouse monoclonal) were purchased from Santa Cruz Biotechnology (CA, U.S.A.), and antibodies against MDM2 (ab38618, rabbit polyclonal), CDK6 (ab3126, mouse monoclonal), and GADD45A (ab180768, rabbit polyclonal) were purchased from Abcam (Cambridge, U.K.). Finally, the membranes were incubated with a horseradish peroxidase-conjugated secondary antibody (Santa Cruz Biotechnology, CA, U.S.A.; sc-2004, goat anti-rabbit IgG-HRP; sc-2005, goat anti-mouse IgG-HRP), and the immunoactivity was detected using ECL-Plus kit (Amersham Biosciences, Piscataway, NJ, U.S.A.).

### Packaging of shSTIM1 lentivirus

ShRNA target sequence (5′-GGGAAGACCTCAATTACCA-3′) for STIM1 gene (NM_003156) and a non-silencing sequence (5′-GCGTCCTCATACCAGGATAAA-3′) were designed. shRNA constructs were synthesized and cloned into the pGCSIL-GFP vector by GeneChem Corporation. The pGCSIL-shRNA-GFP, pHelper1.0, and Helper2.0 were mixed and transfected into 293T cells according to the instructions of Lipofectamine™ 2000 (Invitrogen, Carlsbad, CA, U.S.A). After 48 h transfection, lentiviral particles were harvested from the cell culture medium and then filtered through 0.45 µm PVDF membranes. The cells were infected with lentivirus for 48 h and then the RNA and protein were isolated.

### High-content screening for cell proliferation assay

High-content screening (HCS) was used to measure cell growth. After 72 h infection with shCtrl lentivirus or STIM1-shRNA lentivirus, Tca-8113 cells were reseeded into 96-well plates (2000 cells/well) at 37°C containing 5% CO_2_ for 5 days. ArrayScan™ HCS software (Cellomics Inc. Pittsburgh, PA, U.S.A.) was used to analyze cell proliferation of each well every day, which could automatically identify and count the stained cells in each individual cell. Images were acquired for each fluorescence channel by using suitable filters and 20× objective. Each experiment was performed in triplicates.

RETRACTED

### Colony formation assay

After infecting with NC lentivirus or STIM1-shRNA lentivirus, cells were seeded in six-well plates at a density of 800 cells per well, and culture medium was changed every 2 days. Colonies were checked after incubation for 14 days at 37°C. Then, adherent cells were washed twice with PBS and fixed with 4% paraformaldehyde (Sinopharm, Shanghai, China) for 30 min. After stained with Giemsa solution (Dingguo Bio, Shanghai, China) for 10 min, the colonies were washed twice with double distilled water. All experiments were performed in triplicate.

### Apoptosis assay

Annexin V-APC apoptosis detection kit (Ebioscience, San Diego, CA, U.S.A.) was used to analyze cell apoptosis by staining viable cells according to the manufacturer’s protocol. Briefly, after 3 days infected with NC lentivirus or STIM1-shRNA lentivirus, Tca-8113 cells were harvested, washed with PBS, and resuspended using staining buffer at a final density of 1 × 10^6^–1 × 10^7^/ml. Then, 5 μl of Annexin V-APC was added into 100 μl of the above cell suspension and the mixture was incubated at room temperature for 15 min, finally subjected to flow cytometry (FACSCalibur, Becton-Dickinson, U.S.A.).

### Cell cycle assay

Cell cycle progression was determined by propidium iodide (PI, Sigma–Aldrich, Co., LLC, St. Louis, MO, U.S.A.) staining using a flow cytometer. In brief, cells were infected with NC lentivirus or STIM1-shRNA lentivirus. After incubation for 96 h, cells were seeded in six-well culture plates and cultured to 80% confluence. Next, cells were fixed with 70% cold ethanol at 4°C overnight. Then, cells were rehydrated and washed twice with ice-cold PBS, and incubated with 10 mg/ml RNase (Fermentas, Shanghai, China) at 37°C. Then, cell cycle was monitored by using PI staining of nuclei. Cell cycle was analyzed by FACS on a flow cytometry (FACS Calibur, Becton Dickinson, San Jose, CA, U.S.A.).

### Microarray

Total RNA from tongue squamous carcinoma cells was extracted using Trizol reagent (Invitrogen). NanoDrop 2000 (Thermo Fisher Scientific, Wilmington, DE, U.S.A.) and Agilent Bioanalyzer 2100 (Agilent, Palo Alto, CA, U.S.A.) were used to detect the RNA quantity and quality. Affymetrix human GeneChipprimeview (Affymetrix, Santa Clara, CA, U.S.A.) was used for microarray processing to determine gene expression profile according to the manufacturer’s instructions. Significantly different genes between Tca-8113 cells treated with shCtrl and shSTIM1 were identified depending on the following criteria: *P*<0.05 and the absolute fold change >1.5. Pathway enrichment analysis was performed for all significantly different genes based on KEGG and BIOCARTA pathway databases.

RETRACTED

### Statistical analysis

The statistical analyses were performed using SPSS 16.0 software (SPSS, Inc., Chicago, IL, U.S.A.). The data shown are presented as the mean ± S.E.M. of at least three independent repeats, if no any other statements. Student’s *t*-tests were used to analyze the differences between two groups. A probability value of less than 0.05 was considered significant.

## Results

### STIM1 expression in human tongue squamous carcinoma cells

To investigate the STIM1 expression pattern in human tongue squamous carcinoma cells, we tested the STIM1 mRNA level in two tongue squamous carcinoma cell lines, Tca-8113 and CAL27. As shown in Figure 1A, STIM1 was expressed in the two cell lines. Next, to explore the role of STIM1 in tongue squamous carcinoma, we knocked down STIM1 with lentivirus-mediated shRNA in Tca-8113 cells. As shown in Figure 1B, the infection efficiency was visibly high (>80%) as evidenced by the expression of the reporter gene *GFP*. Significantly, endogenous STIM1 mRNA was significantly reduced in the shSTIM1 group with 71.3%, compared with control group (Figure 1C).

**Figure 1:** STIM1 was expressed and knocked down in human tongue squamous carcinoma cells (**A**) Expression of STIM1 mRNA was measured by qRT-PCR in two tongue squamous carcinoma cell lines, Tca-8113 and CAL27. The relative expression of STIM1 is shown as Δ*C*_T_ (*C*_T_^STIM1 ^−*C*_T_^GAPDH^). (**B**) Representative image showing lentivirus infection in Tca-8113 cells. Tca-8113 cells were infected with shSTIM1 and shCtrl lentivirus for 48 h, and then the efficiency of infection was assessed by light microscopy and fluorescent microscopy at the third day infection. (**C**) Knockdown of STIM1 in Tca-8113 cells. Tca-8113 cells were infected with shSTIM1 and shCtrl lentivirus for 48 h, and then qRT-PCR analysis was performed to analyze the mRNA level of STIM1 in Tca-8113 cells; ***P<0.001.

### STIM1 regulates proliferation and colony formation of human tongue squamous carcinoma cells

Furthermore, to detect the effect of STIM1 on Tca-8113 proliferation, HCS was used to monitor cell growth every day for 5 days. The results showed that STIM1 knockdown decreased the total number of cells (Figure 2A and B), and the cell growth rate was declined approximately 6-fold (Figure 2C).

RETRACTED

**Figure 2:** STIM1 knockdown inhibits Tca-8113 cell proliferation (**A**) Representative images of Tca-8113 cells infected with shCtrl (top) and shSTIM1 (bottom) via multiparametric HCS every day for 5 days. (**B**–**C**) STIM1 knockdown represses cell proliferation of Tca-8113 cells. Tca-8113 cells infected with shCtrl and shSTIM1, and cell number was analyzed everyday by HCS.

Furthermore, we performed colony formation assay to confirm the suppression of tumorigenesis by STIM1 down-regulation. As shown in Figure 3A, suppression of STIM1 expression significantly decreased the colony formation. The number of colonies in the shSTIM1 group was apparently fewer than that in shCtrl group (106 ± 6 compared with 30 ± 2, *P*<0.001, Figure 3B). Taken together, these results suggested that STIM1 was necessary in Tca-8113 cell proliferation.

**Figure 3:** Clonogenic ability was suppressed in Tca-8113 cells by STIM1 knockdown (**A**) Pictures of colony formation by Tca-8113 cells infected with lentivirus expression either shCtrl or shSTIM1 using Giemsa staining on the 14th day. (**B**) Quantitation of clone number formed by Tca-8113 cells infected with lentivirus expression either shCtrl or shSTIM1. The results represent mean ± S.E.M.; ***P<0.001.

### STIM1 regulates cell cycle

It is well known that the cell cycle arrest may affect the cell proliferation. On this context, we investigated whether STIM1 could regulate cell cycle progression by PI/FACS. As expected, down-regulation of STIM1 expression significantly led to G_1_-phase arrest and decreased cell percentage of S phase (Figure 4A and B). As shown in Figure 4B, the cell percentage in G_1_ phase was markedly increased in shSTIM1 group compared with shCtrl group (46.45 ± 0.28% compared with 41.67 ± 0.60%). On the other hand, compared with shCtrl group, cell population of S phase was significantly decreased in shSTIM1 group (47.59 ±1.04% compared with 41.44 ± 0.33%). The G_2_/M phase was not regulated by the STIM1 (Figure 4B). These results indicated that knockdown of STIM1 inhibited tongue squamous carcinoma cells growth partially by inducing cell cycle arrest.

**Figure 4:** Knockdown of STIM1 regulates cell cycle of Tca-8113 cells (**A**) Representative result showing STIM1 knockdown represses cell cycle in Tca-8113 cells. Tca-8113 cells were infected with shCtrl or shSTIM1 lentivirus for 48 h and then flow cytometry was performed to analyze cell cycle. (**B**) STIM1 knockdown induces cell cycle arrest at G_1_ phase. Tca-8113 cells were infected with shCtrl or shSTIM1 lentivirus for 48 h and then flow cytometry was performed to analyze cell cycle; ***P<0.001.

RETRACTED

### STIM1 knockdown induces Tca-8113 cell apoptosis

Resisting apoptosis is essential the tumor cell [9,10]. Hence, we investigated whether STIM1 expression affects apoptosis using Annexin V staining followed by flow cytometry method (Figure 5A). As shown in Figure 5B, STIM1 knockdown markedly increased apoptosis in Tca-8113 cells compared with control group (8.87 ± 0.31% compared with 4.74 ± 0.20%). These results indicated that STIM1 was a determinant of cell apoptosis, which may contribute to the effect of STIM1 on cell proliferation of Tca-8113 cells.

**Figure 5:** STIM1 knockdown induces apoptosis in Tca-8113 cells (**A**) Representative images showing STIM1 knockdown induces apoptosis in Tca-8113 cells. Tca-8113 cells were infected shCtrl or shSTIM1 for 48 h and then cell apoptosis was determined by Annexin V staining and flow cytometry. R3 region indicates the percentage of apoptotic cells. (**B**) Quantitation of cell apoptosis induced by knockdown of STIM1 in (A); ***P<0.001.

### Knockdown of STIM1 disrupts multiple critical pathways in human tongue squamous carcinoma cells

The above results showed that STIM1 was critical for tumorigenesis in human tongue squamous carcinoma cells Tca-8113. However, the mechanisms underlying STIM1-mediated phenotypes and the downstream pathways were still unknown. Therefore, global gene expression profile of Tca-8113 cells infected with lentivirus expressing either shCtrl or shSTIM1 was examined using microarray platform. We identified 1841 genes with significant difference (fold change >1.5 and *P*<0.05), including 833 up-regulated genes and 1008 down-regulated genes (Figure 6A). Then, KEGG pathway analysis was performed and the differentially expressed genes were enriched in ten pathways. As expected, two pathways, pathways in p53 and MAPK were significantly enriched in cells with STIM1 knockdown (Figure 6B). Given that STIM1 suppression can block the cell cycle in Tca-8113 cells (Figure 4A and B), we focussed on the cell cycle pathway. As shown in Figure 6C, the expression of cell cycle-related genes, such as cyclin family, were regulated by knockdown of STIM1, suggesting that STIM1 was necessary for normal cell cycle progression. To confirm these results, we selected three key genes of p53 (MDM2, CKD6, and GADD45A) to confirm the gene expression that induced by STIM1 using Western blot. As expected, knockdown of STIM1 significantly affected the protein level of MDM2, CDK6, and GADD45A (Figure 6D). These results indicated that STIM1 inhibited the cell proliferation mainly by blocking cell cycle progression via regulating p53 pathway.

RETRACTED

**Figure 6:** Knockdown of STIM1 disruption multiple critical pathways in human tongue squamous carcinoma cells (**A**) Heatmap representation of 1841 genes (833 genes up-regulated and 1008 genes down-regulated) with differential expressions in Tca-8113 cells infected with lentivirus expressing either shCtrl or shSTIM1 (criteria: *P*<0.05, fold change >1.5). (**B**) Functional pathway enrichment of differential genes was analyzed based on KEGG and BIOCARTA databases. (**C**) Interactional network was constructed between STIM1 and genes involved in KEGG pathway cell cycle. Green circles represent down-regulated genes, red circles represent up-regulated genes and genes of gray circles represent no expression changing. (**D**) STIM1 regulates the expression of MDM2, CDK6, and GADD45A. Tca-8113 cells were infected with shCtrl or shSTIM1 for 48 h and then Western blot was performed to analyze the expression of MDM2, CDK6, and GADD45A.

## Discussion

In the present study, we investigated the function of STIM1 in human OSTCC. Using loss-of-function strategy, we demonstrated that STIM1 promoted the growth of human OTSCC cells by regulating apoptosis and cell cycle. We showed that STIM1 knockdown inhibited cellular proliferation and colony formation of OTSCC cells. The mechanism of our study indicated that STIM1 knockdown repressed cell cycle to enter M phase and induced apoptosis in OSTCC cells. Furthermore, our microarray data showed that STIM1 controlled the p53 and MAPK pathways. Our molecular analysis also confirmed that STIM1 regulated the protein level of MDM2, CDK4, and GADD45A.

STIM1 is an ER Ca^2+^ sensor that triggers the SOCE activation. Recently, STIM1 has recently been implicated in cancer progression of different types of cancer. In prostate cancer, STIM1 accelerates cell senescence in a remodeled microenvironment but enhances the epithelial-to-mesenchymal transition [6]. STIM1-mediated SOCE is also required for HIF-1 accumulation in hypoxic hepatocellular carcinoma via activation of Ca^2+^/calmodulin-dependent protein kinase II and p300. Administration of the HIF inhibitor, YC-1, or knockdown of HIF1α significantly diminishes hypoxia-enhanced STIM1 and suppresses tumorigenesis [11]. Enhanced expression of STIM1 promotes CRC cell metastasis *in vitro* and *in vivo* by inducing epithelial-to-mesenchymal transition or COX-2 expression [7,12]. Our previous findings demonstrated that STIM1 promotes cell cycle and survival to facilitate tumor growth of human hypopharyngeal carcinoma [8]. We found here that STIM1 also essentially participates in the development of human OSTCC. Knockdown of STIM1 expression inhibited the proliferation of Tca-8113 cells. In addition, the colony formation ability of Tca-8113 cells was also repressed by STIM1 knockdown. These findings indicate that STIM1 is essentially involved in human OTSCC.

RETRACTED

Further mechanistic studies showed that knockdown of STIM1 repressed cell cycle at G_1_ phase. The percentage of cells in G_1_ phase was significantly increased whereas the percentage of cells in S phase is reduced. However, the percentage of cells at G_2_/M phase was not affected by STIM1. Interestingly, our previous work indicated that knockdown of STIM1 reduced the percentage of G_2_/M phase [8]. Further work is needed to elucidate how these differences exist in two different kinds of cancer. In addition, we also found that STIM1 regulated cell survival. Knockdown of STIM1 induced a significant increase in apoptotic cells in Tca-8113 cells, which is consistent with the function of STIM1 in human hypopharyngeal carcinoma [8], pancreatic adenocarcinoma [13], and non-small cell lung cancer [14]. In contrast, STIM1 knockdown did not alter proliferation or apoptosis, but promoted cell adhesion and inhibited migration and invasion in the gastric cancer cells [15], indicating that STIM1 plays different roles in different cancers.

We also performed microarray and bioinformatics analysis which indicated that the top three pathways affected by STIM1 were cell cycle, MAPK, and p53 pathways. Other pathways include WNT, GPCR, and Neurotrophin pathways. We also performed Western blotting and confirmed that STIM1 knockdown inhibited the expression of MDM and CDK6, two proteins that are involved in the p53 pathway. P53 activates MDM, which in turn could reduce the stability of p53 and inhibits its activity, p53 also inhibits the activity of CDK6 by promoting p21 [16,17]. In addition, STIM1 knockdown promoted the expression of GADD45A, a p53 downstream stress-inducible gene. P53 binds GADD45A promoter and promotes GADD45A transcription to regulate base excision repair [18,19]. Therefore, the p53 pathway was involved in the function of STIM1 in Tca-8113 cells. The MAPK pathway was also significantly affected by STIM1. In consistent, SOCE induced by protease-activated receptor-1 mediates STIM1 protein phosphorylation to inhibit SOCE in endothelial cells through p38β mitogen-activated protein kinase (MAPK) [20]. Interestingly, a previous report of STIM1 knockdown did not alter the expression or phosphorylation of MAPK or extracellular signal-regulated kinase (ERK) in gastric cancer [15], indicating that STIM1 regulates different pathways in different cancer types, which may account for the different roles of STIM1 in different cancers. However, further works are needed to elucidate how STIM1 regulates the p53 and MAPK pathways to modulate cell survival and growth. STIM1 is located in ER and acts as a key component of SOCE. STIM1 plays a dual role as an ER Ca^2+^ receptor and an SOCE exciter. STIM1 senses the ER Ca^2+^ concentration via a luminal, N-terminal located, canonical EF hand [4,5]. Therefore, it is also interesting to investigate whether Ca^2+^ influx is involved in the effects of STIM1 on growth, cell cycle, and apoptosis of human tongue squamous carcinoma cells.

RETRACTED

In conclusion, we identify STIM1 as an oncogenic protein in human OTSCC. Our findings indicate that STIM1 promotes cell cycle, cell survival, and growth by regulating the p53 and MAPK pathways. Therefore, OTSCC may serve as a prognostic factor and therapeutic target in human OTSCC.

## Abbreviations

APC: Adenomatous polyposis coli
CDK4: cyclin-dependent kinase 4
COX-2: Cyclooxygenase-2
CRC: colorectal cancer
ER: endoplasmic reticulum
GAPDH: Glyceradldehyde-3-3phosphate dehydrogenase
GADD45A: growth arrest and DNA damage inducible α
GPCR: Guanosine-binding Protein Gcoupled Receptor
HCC: hypoxic hepatocarcinoma
HCS: high-content screening
HIF: hypoxia-inducible factor
KEGG: Kyoto Encyclopedia of Genes and Genomes
MAPK: mitogen-activated protein kinase
MDM2: Transformed mouse 3T3 cell double minute 2
M-MLV: Moloney murine leukemia virus
NC: Negative Control
OTSCC: oral tongue squamous cell carcinoma
PI: propidium iodide
qRT-PCR: quantitative real-time PCR
RIPA: Radio-Immunoprecipitation Assay
SOCE: store-operated calcium entry
STIM1: stromal interaction molecule 1
SYBR: Synergy Brands
YC-1: RNA binding motif single stranded interacting protein 1
